# Effectiveness and Safety of Saccharomyces Boulardii for the Treatment of Acute Gastroenteritis in the Pediatric Population: A Systematic Review and Meta-Analysis of Randomized Controlled Trials

**DOI:** 10.1155/2022/6234858

**Published:** 2022-09-20

**Authors:** Hongbo Fu, Jinrong Li, Xunhua Xu, Caihuai Xia, Yajuan Pan

**Affiliations:** ^1^Department of Emergency, Haikou Maternal and Child Health Hospital, Haikou 570203, China; ^2^Department of Pediatrics, Haikou Hospital of Traditional Chinese Medicine, Haikou 570216, China; ^3^Department of Pediatrics, Wenchang City People's Hospital, Wenchang 571300, China

## Abstract

**Objective:**

To explore the efficacy and safety of Saccharomyces boulardii for the treatment of acute gastroenteritis in children aged under 5.

**Methods:**

Two independent researchers retrieved literature from PubMed, OVID, Embase, ScienceDirect, and other databases, followed by extracting indicators of the primary endpoints. Cochrane Q test and *I*^2^ statistics were used to evaluate interstudy heterogeneity. The relative risk (RR) and mean difference (MD) of related indicators were calculated and combined using the random- or fixed-effect model, as appropriate. Furthermore, the funnel plot and Egger's test were used to evaluate the publication bias. A two-sided *P* < 0.05 denoted statistical significance.

**Results:**

10 articles were included in this meta-analysis, with a total of 1282 children having acute gastroenteritis. The use of Saccharomyces boulardii in children with acute gastroenteritis could effectively shorten diarrhea duration (MD = 19.70, 95% CI: -24.87, 14.52) and reduce the length of hospital stay (MD = −0.91, 95% CI: -1.28, -0.54). Compared with the control group, the RR of continued diarrhea was significantly lower in the treatment group after 1 day treatment (RR = −0.31, 95% CI: 0.59, 0.03) and 3 days treatment (RR = 0.52, 95% CI: 0.41, 0.66). In addition, treatment with Saccharomyces boulardii reduced the average number of diarrhea after 3 days of treatment by about 1.03 (MD = −1.03, 95% CI: -1.53, -0.53). There were no adverse drug reactions in both groups.

**Conclusion:**

The use of probiotic Saccharomyces boulardii can significantly improve the symptoms of diarrhea in children with acute gastroenteritis and reduce the duration of diarrhea symptoms and the time of hospitalization. Meanwhile, the RR of continued diarrhea in children after 1 and 3 days of Saccharomyces boulardii treatment and the frequency of diarrhea after 3 days of Saccharomyces boulardii treatment were decreased. It is also safe and does not increase the incidence of adverse drug reactions.

## 1. Introduction

Acute gastroenteritis is a gastrointestinal mucosal inflammation characterized by diarrhea, vomiting, nausea, and abdominal pain. Pediatric gastroenteritis is mainly caused by norovirus and rotavirus [1, 2]. Although acute gastroenteritis in children is a self-limiting disease and oral rehydration therapy (ORT) can significantly shorten the course of the disease [3–5], there are still clinical challenges in the treatment of children with dehydration and vomiting symptoms in terms of ORT therapy failure and hospitalization [2]. Some studies have shown that not using ORT therapy or failure of ORT therapy significantly increases the risk of dehydration, electrolyte imbalance, intravenous infusion, and hospitalization in children with acute gastroenteritis, especially younger children [6]. Although acute gastroenteritis is treatable and preventable, it is still one of the major factors leading to the “death burden” in children aged 5 years and under. Death in children with acute gastroenteritis are most commonly related to severe dehydration [7].

A large number of children worldwide suffer from acute gastroenteritis every year, of which approximately 150000-250000 died [8]. It is estimated that the incidence of acute gastroenteritis in children under 5 years of age in developing countries is about 3-5 cases per person per year [9, 10]. The incidence of acute gastroenteritis-related death in children under 5 years is about 200 thousand [11] in developing countries, whereas it is about once per person per year in developed countries [12].

Several clinical guidelines suggest that probiotics with promising efficacy and safety should be used as adjuvant treatment for liquid therapy of acute gastroenteritis [13–15]. Although Listeria rhamnosus and Saccharomyces boulardii were the two most used probiotics in clinical practice and recommended by the guidelines, the literature on Listeria rhamnosus is insufficient, and their efficacy in the treatment of acute gastroenteritis remains controversial, which is probably related to inconsistent study conclusions and methodological defects. Increasing randomized controlled trials have shown that Saccharomyces boulardii can effectively shorten the duration of diarrhea in patients with acute gastroenteritis [16]. Therefore, this study explored the safety and effectiveness of Saccharomyces boulardii in treating children with acute gastroenteritis through systematic review and meta-analysis to provide more evidence for the role of probiotics for pediatric acute gastroenteritis and the prevention of dehydration and electrolyte disorders.

## 2. Methods

### 2.1. Literature Search

This study used Medical Subject Headings (MESH) as search terms in PubMed, Embase, ScienceDirect, OVID, and other databases for literature retrieval. The search keywords were (“Infant”[Mesh Terms] OR “children” OR “pediatrics” OR “adolescent”) AND (“Probiotics”[Mesh Terms] OR “Saccharomyces boulardii”) AND (“diarrhea” OR “vomiting” OR “Dehydration” OR “diarrhea∗” OR “emesis” OR “gastroenteritis”).

### 2.2. Literature Screening

The inclusion criteria were: (1) placebo-controlled randomized controlled trial (RCT); (2) children with confirmed acute gastroenteritis as the study population; (3) children aged under 5; (4) Saccharomyces boulardii used for treatment; (5) study main endpoints included at least one of the following six categories: duration of diarrhea, length of hospital stay, stopping diarrhea within 1 day, stopping diarrhea within 3 days, the number of diarrhea after treatment, and the occurrence of adverse drug reaction events.

Literature exclusion criteria: (1) study population limited to a special population, such as people with immune deficiency or those with concomitant gastrointestinal diseases, such as necrotizing colitis, Crohn's disease; (2) studies with subject overlap; (3) sample size of the interventional group or control group less than 20; (4) nonoriginal articles, such as comments, academic conferences, reviews, and case reports. No restrictions of the pathogens that cause acute gastroenteritis were applied in this study.

### 2.3. Document Data Sorting and Evaluation

The following data were screened and extracted from the literature by Fu and Li (Table 1): study type (open trial or double-blind trial), number of subjects in the control group and the interventional group, demographic characteristics, duration of diarrhea, duration of hospitalization, continuous diarrhea for 1 day after treatment, continuous diarrhea for 3 days after treatment, diarrhea frequency, and incidence of adverse drug reactions. Study quality was evaluated with the Newcastle Ottawa Scale (NOS), with scores below 5, 5-7 and ≥8 denoted low-, medium-, and high-quality publications. Controversies between the 2 investigators were settled by discussion and consultation with the third researcher.

### 2.4. Statistical Methods

The STATA17.0 (SE) software was employed for statistical analysis. The observed primary clinical endpoint for categorical and continuous variables were expressed by relative risk (RR) and mean ± standard deviation, respectively. The random- and fixed-effect model were used in the presence of significant (*I*^2^ > 50%) and nonsignificant interstudy heterogeneity, respectively. Interstudy heterogeneity was assessed by the Cochran's Q test. In the absence of interstudy heterogeneity (*P* > 0.05 and *I*^2^ < 50%), the fixed-effect model was used. Otherwise, the random-effect model was used. The funnel plot, Egger's and Begg's tests were utilized to evaluate publication biases. A two-sided *P* value less than 0.05 denoted statistical significance.

## 3. Results

### 3.1. Search Results and Literature Characteristics

A total of 188 relevant literatures were generated, of which 10 studies were included in the meta-analysis according to the established inclusion and exclusion criteria. The detailed process of literature retrieval and screening was presented in Figure 1. All the included literatures were clinical RCTs that included 1282 children in total. Among the 10 studies, 8 reported diarrhea duration in children with acute gastroenteritis after the use of Saccharomyces boulardii, 5 reported hospitalization time, 4 evaluated the diarrhea frequency on the third day after treatment, 6 reported the diarrhea lasting for one day after treatment, and 7 reported persistent diarrhea for 3 days after treatment. According to the risk-of-bias assessment proposed by Cochrane, only 3 included publications described the grouping concealment and blind method of randomized grouping, which was considered to have a low risk of bias, and the rest of the literature had a moderate- to high-risk of bias. NOS scores ranged from 4 to 8, including 3 high-quality, 4 medium-quality, and 3 low-quality literature.

### 3.2. Duration of Diarrhea

A total of 1051 children in 8 studies were included for the evaluation of diarrhea duration. The heterogeneity test results were *H*^2^ = 6.99, *I*^2^ = 85.70%, *P* < 0.001, indicating a high degree of heterogeneity. Therefore, the random-effect model based on the restricted maximum likelihood method was used to combine the mean difference. Meta-analysis (Figure 2) showed that compared with placebo, the use of Saccharomyces boulardii significantly reduced the duration of diarrhea in children with acute gastroenteritis (Mean difference = 19.70, 95% CI: -24.87, 14.52, *P* < 0.001). The funnel plot showed points on both sides in an inverted funnel shape, and two studies were outside the confidence interval. Eegg's test that was performed on the included studies indicated absence of obvious publication bias (*Z* = 0.50, *P* = 0.617, Figure 3).

### 3.3. Length of Hospital Stay

A total of 755 children from 5 literatures were included. Moderate heterogeneity (*H*^2^ = 4.01, *I*^2^ = 75.05%, *P* < 0.001) was noted, for which the random-effect model was used. Compared with the control group, the use of Saccharomyces boulardii significantly reduced length of hospitalization in children with acute gastroenteritis by about 0.91 days (Mean difference = −0.91, 95% CI: -1.28, -0.54, *P* < 0.001, Figure 4). The funnel plot and Eegg's test indicated no obvious publication bias (*Z* = −1.86, *P* = 0.108, Figure 5).

### 3.4. Diarrhea for 1 Day after Treatment

A total of 1049 subjects from 7 studies were included. The random-effect model was used since the interstudy heterogeneity was modest (*H*^2^ = 2.84, *I*^2^ = 64.85%, *P* < 0.005). The result (Figure 6) indicated that Saccharomyces boulardii significantly reduced the risk of persistent diarrhea within 1 day after treatment in children with acute gastroenteritis (RR = 0.70, 95% CI: 0.49, 1.00, *P* = 0.01). The funnel plot shows that the points are distributed on both sides, within the confidence interval, in an inverted funnel shape, but one study is outside the confidence interval. No obvious publication bias was suggested by the Eegg's test (*Z* = −0.9, *P* = 0.548, Figure 7).

### 3.5. Diarrhea Lasting for 3 Days after Treatment

Seven studies with 1049 children in total were used for meta-analysis. Minimal heterogeneity was noted (*H*^2^ = 1.00, *I*^2^ = 0.00%, *P* = 0.77), for which the fixed-model was utilized. The results of the meta-analysis showed that compared with the control group, the use of Saccharomyces boulardii could reduce the risk of 3-day continuous diarrhea in children with acute gastroenteritis after treatment (RR = 0.52, 95% CI: 0.41, 0.66, *P* < 0.001), as shown in Figure 8. No publication bias was found by the funnel chart (Figure 9).

### 3.6. Diarrhea Frequency after Treatment (the Third Day)

A total of 519 patients in 5 studies with minimal interstudy heterogeneity (*H*^2^ = 1.09, *I*^2^ = 7.87%, *P* = 0.49) were meta-analyzed with the fixed-effect model. The results showed that Saccharomyces boulardii significantly reduced the frequency of diarrhea in children with acute gastroenteritis after treatment by about 1.03 times (Mean difference = −1.03, 95% CI: -1.53, -0.53, *P* < 0.001, Figure 10). The funnel chart (Figure 11) suggested no publication bias.

## 4. Discussion

Probiotics refer to the microbiota that can colonize and survive in the host and play a beneficial role in health [27]. In recent years, the role of probiotics in health promotion, health protection, disease treatment, and regulation of intestinal flora has attracted increasing attention [28, 29]. In vitro and animal model experiments have shown that probiotics can exert their biological role by competing with pathogenic bacteria for nutrition and binding sites, producing antibacterial substances, providing nutrients for colonic epithelial cells, and reducing intestinal permeability [30, 31]. Other mechanisms related to treating acute gastroenteritis in children included altered gene expression of epithelial cells, increased activity of phagocytes and natural killer cells, and elevated level of immunoglobulin A in saliva and feces [30, 31]. Emerging evidence support that probiotics can also regulate human immune responses, in which the dendritic cells and toll-like receptor molecules played a pivotal role. These cells or molecules regulate the production of endogenous immune peptides by receiving structural lipopolysaccharides, glycopeptide molecules, and CpG DNA from probiotics and conducting biological conversion on them [32]. Specifically, Saccharomyces boulardii produced 54 KD protease that can hydrolyze clostridium difficile endotoxin and their corresponding binding sites on intestinal cells, and stimulated production of specific IgG and IgA in the meantime. In addition, some studies have found that probiotics can stimulate the production of anti-inflammatory factors (e.g., interleukin [IL]-10 and IL-4) and inhibit proinflammatory factors tumor necrosis factor- *a* and interferon- *γ*, thus promoting the digestive tract mucosa to produce specific anti-rotavirus secretory IgA and regulating the mucosal immune response to pathogens [33].

In a 2010 Cochrane meta-analysis [34], Allen et al. showed that the use of probiotics could reduce the diarrhea time of children with acute gastroenteritis (-25 h, 95% CI: -16 h, -34 h); the proportion of diarrhea lasting four days or more (RR 0.41, 95%ci: 0.32, 0.53) was comparable with the results of this study. Szajewska et al. found through meta-analysis that Lactobacillus rhamnosus could also shorten the diarrhea time of children with acute gastroenteritis by about 1.05 days (95% CI: -1.7, -0.4), and this effect was more significant in the high-dose group. Of note, the main population of this study was Caucasians. Considering the differences in common colonized flora in the gastrointestinal tract between Chinese and Western population, the conclusions of this study might not be extrapolated to the Chinese population [35]. Previous meta-analyses indicated positive effects of probiotics for treating acute gastroenteritis in children. This evidence-based medical evidence has prompted many institutions to recommend promoting the daily use of probiotics in pediatric inpatients [36]. However, some scholars still believe that the evidence for the widespread use of probiotics in patients with acute gastroenteritis is still weak, especially in outpatients [37]. Furthermore, methodological defects of the RCTs included in the above meta-analysis was also a concern. For example, although 63 literatures were included in the meta-analysis by Allen et al., only 10 met all the methodological requirement for RCTs.

This study suffers from several limitations: (1) Although all the included literature in this study was of medium- or high-quality, the risk of bias, including the use of grouping concealment, randomization, and the selection of blind methods, can not be eliminated. Some literature did not use intention-to-treat analysis, leading to the partial deletion of the final data set; (2) Not all the included RCTs provided the calculation process of sample size. Hence, it was unclear whether the research results had sufficient statistical power to prove their reliability; (3) The wide confidence interval of some endpoint indexes increased the uncertainty of statistical inference; (4) Only 10 literature were included in this paper, and some outcome indicators were less than 10. It is difficult to distinguish the degree of symmetry in the funnel plot evaluation of publication offset, so we combined Egger's and Begg's tests for evaluation. (5) Extensive rotavirus vaccination in some developed countries might lead to changes in the epidemiology of acute gastroenteritis, since rotavirus-associated acute gastroenteritis has been demonstrated to benefit most from probiotics. A subgroup analysis of different disease prototypes was unfeasible in this study since few reported the etiology of acute gastroenteritis; (6) Criteria and clinical practices for hospitalization in children with acute gastroenteritis may differ and introduce bias to this study.

In conclusion, this study showed that the use of Saccharomyces boulardii in children with acute gastroenteritis can significantly shorten the time of hospitalization and diarrhea, and no adverse drug reactions have been observed. It provides some theoretical support for the treatment of acute gastroenteritis in children.

## Figures and Tables

**Figure 1:** Prism flow chart. Process of screening for literature inclusion and exclusion.

**Figure 2:** Forest map of the duration of acute gastroenteritis diarrhea in children treated with Saccharomyces boulardii.

**Figure 3:** Funnel chart of the duration of acute gastroenteritis diarrhea in children treated with Saccharomyces boulardii.

**Figure 4:** Forest chart of hospitalization time in children with acute gastroenteritis treated with Saccharomyces boulardii.

**Figure 5:** Funnel chart of hospitalization time in children with acute gastroenteritis treated with Saccharomyces boulardii.

**Figure 6:** Forest chart of continuous diarrhea for 1 day in children with acute gastroenteritis treated with Saccharomyces boulardii.

**Figure 7:** Funnel chart of continuous diarrhea for 1 day in children with acute gastroenteritis treated with Saccharomyces boulardii.

**Figure 8:** Forest chart of diarrhea for 3 days in children with acute gastroenteritis treated with Saccharomyces boulardii.

**Figure 9:** Funnel chart of the observation results of Saccharomyces boulardii on the 3-day continuous diarrhea after the treatment of acute gastroenteritis in children.

**Figure 10:** Forest chart of diarrhea frequency on the third day after treatment in children with acute gastroenteritis treated with Saccharomyces boulardii.

**Figure 11:** Funnel chart of diarrhea frequency on the third day after treatment in children with acute gastroenteritis treated with Saccharomyces boulardii.

**Table 1:** Characteristics of 12 included literatures.

Author	Study design	Sample size		Age range	Duration of diarrhea (h)		Duration of hospitalization (days)		Persistency of diarrhea on day 1		Persistency of diarrhea on day 3		Diarrhea frequency on day 3		Adverse event	
		Intervention	Control		Intervention	Control	Intervention	Control	Intervention	Control	Intervention	Control	Intervention	Control	Intervention	Control
Das et al. [17]	RCT	30	30	3 months to 5 years	60(51-67)	89(68-95)	3.18 ± 0.58	3.8 ± 0.71	3	10	1	4	NA	NA	NA	NA
Riaz et al. [18]	RCT	54	54	3 months to 5 years	49.55(25.82-73.27)	66.34(27.07,95.81)	NA	NA	13	21	10	15	15.28 ± 11.71	15.92 ± 13.43	NA	NA
Dinleyici et al. [19]	RCT	220	143	4 months to 4 years	60.4 (37.3-83.5)	78.4(57.5-99.3)	4.6 ± 1.72	6.12 ± 1.71	200	130	69	82	NA	NA	NA	NA
Billoo et al. [20]	RCT	50	50	2 months to 12 years	82(45.3-99.2)	92(81.3-112.1)	NA	NA	10	9	3	5	2.8 ± 3.05	4.4 ± 3.05	NA	NA
Cetina-sauri et al. [21]	RCT	65	65	9 months to 20 months	NA	NA	NA	NA	10	19	8	14	2.53 ± 1.78	3.63 ± 2.53	NA	NA
Hafeez et al. [22]	RCT	50	51	3 months to 60 months	NA	NA	NA	NA	NA	NA	NA	NA	4.29 ± 3.07	5.73 ± 3.07	NA	NA
Villarruel et al. [23]	RCT	44	44	3 months to 2 years	147.84(48-312)	112.8(48-240)	NA	NA	22	30	9	23	NA	NA	NA	NA
Kurugöl et al. [24]	RCT	100	100	3 months to 7 years	112.8(50.4-172.8)	132(55.2-208.8)	2.9 ± 1.2	3.9 ± 1.5	18	38	8	24	NA	NA	NA	NA
Grandy et al. [25]	RCT	25	27	1 months to 23 months	58(18-92)	84.5(23.4-112.4)	3.16 ± 1	3.72 ± 2.43	NA	NA	NA	NA	NA	NA	NA	NA
Bhat et al. [26]	RCT	40	40	6 months to 5 years	41.68 ± 10.84	57.65 ± 26.31	2.72 ± 0.42	3.37 ± 1.1	NA	NA	NA	NA	2.6 ± 1.28	3 ± 2.5	NA	NA

## Data Availability

The data used to support the findings of this study are included within the article.
